The article "Analysis of Antiapoptosis Effect of Netrin-1 on Ischemic Stroke and Its Molecular Mechanism under Deleted in Colon Cancer/Extracellular Signal-Regulated Kinase Signaling Pathway" was retracted in 2024. Reasons: signs of a paper mill; compromised peer review; unreliable results or conclusions.

# Analysis of Antiapoptosis Effect of Netrin-1 on Ischemic Stroke and Its Molecular Mechanism under Deleted in Colon Cancer/Extracellular Signal-Regulated Kinase Signaling Pathway

**DOI:** 10.1155/2020/8855949

**Published:** 2020-11-14

**Authors:** Kai Wang, Liangqun Rong, Xiu'e Wei, Qingxiu Zhang

**Affiliations:** Department of Neurology, Second Affiliated Hospital of Xuzhou Medical University, Xuzhou 221006, China

## Abstract

To analyze the regulatory effect of Netrin-1 in ischemic stroke and its influence on Deleted in Colon Cancer (DCC)/Extracellular Signal-regulated Kinase (ERK) signaling pathway, 20 male rats were selected to construct the rat model of middle cerebral artery occlusion (MCAO), 10 normal rats were selected as healthy controls (Normal Saline (NS)), and they were divided into the MCAO+Netrin-1 group, MCAO group, and NS group according to different treatment schemes. The positive expression of Netrin-1 was detected by immunostaining, magnetic resonance imaging (MRI) was adopted to detect the percentage of rat cerebral infarct volume in the cerebral hemispheres, and Modified Neurological Severity Score (mNSS) was adopted to evaluate postoperative neurological function in rats. Besides, a tunnel staining experiment was applied to detect the apoptosis rate of rat neurons, the sticker removal test was applied to evaluate the postoperative sensory function of rats, and fluorescence staining was adopted to detect the expression of DCC and ERK in rats. The results showed that the percentage of cerebral infarction volume in the cerebral hemispheres of the MCAO+Netrin-1 group was higher than that of the MCAO and NS groups (*P* < 0.05); in the MCAO+Netrin-1 group, the MCAO mNSS scoring and the time spent in the sticker removal test were lower than the MCAO group (*P* < 0.05); the apoptosis rate of rats in the MCAO+Netrin-1 group was lower than that in the MCAO group (*P* < 0.05); the average fluorescence intensity of DCC and p-ERK in the MCAO+Netrin-1 group was higher than that in the MCAO group (*P* < 0.05); the average fluorescence intensity of p-ERK in the MCAO+Netrin-1 group was higher than that in the MCAO group (*P* < 0.05). In short, Netrin-1 can effectively reduce the brain tissue damage in rats with ischemic stroke, improve the nerve function and sensory function of rats, and inhibit neuronal cell apoptosis. Netrin-1 can promote DCC expression and ERK phosphorylation, and the EPK signaling pathway may be involved in the antiapoptotic effect of Netrin-1.

## 1. Introduction

Ischemic stroke is a common cerebrovascular disease, which is brain tissue necrosis caused by the stenosis or occlusion of the blood supply arteries of the brain (carotid and vertebral arteries), or insufficient blood supply to the brain. Stroke occurs more frequently in the elderly over 60 years old, and it is also the second leading cause of death in this group of people, with a high disability and mortality rate [1–3]. As the world's aging process accelerates, it is estimated that by 2050, there will be about 1.5 billion people over 65 years of age, and the incidence of stroke will also increase significantly [4]. Symptoms such as dizziness, diplopia, black eyes, numbness of the contralateral limb, weakness, and sensory disturbance may occur when the disease occurs. In severe cases, there may even be hemiplegia, hemianopia, aphasia, sensory disturbance, and disturbance of consciousness, and in severe cases, it threatens the lives [5]. Clinical observations have found that a variety of signal pathways may be activated when the ischemic stroke occurs, causing different degrees of damage to the brain tissue and then leading to neuronal cell apoptosis [6]. Therefore, the key point for the treatment of ischemic stroke is the protection of neurons in the ischemic environment.

The article "Analysis of Antiapoptosis Effect of Netrin-1 on Ischemic Stroke and Its Molecular Mechanism under Deleted in Colon Cancer/Extracellular Signal-Regulated Kinase Signaling Pathway" was retracted in 2024. Reasons: signs of a paper mill; compromised peer review; unreliable results or conclusions.

Netrin receptors are a family of extracellular proteins that can regulate cell migration or survival after individual development and maturation. As the first member of the Netrin family, Netrin-1 can guide the development of the nervous system as an axon guide molecule in the nervous system [7, 8]. Netrin-1 can also bind to different types of receptors, such as the receptor for DCC, the Unc5 family, and neogenin [9]. Among them, the DCC receptor is an extracellular domain composed of more than 1000 amino acids, which can promote the chemotaxis of axons when combined with Netrin-1. Extracellular signal-regulated kinase 1/2 (ERK1/2) is one of the signal pathways of the mitogen-activated protein kinase family. Studies have found that the phosphorylation of ERK1/2 in patients with ischemic stroke will greatly increase. Therefore, many scholars believe that ERK1/2 may also be involved in the progression of ischemic stroke, but the specific regulatory mechanism is still unclear [10–12]. Therefore, this study intended to use Netrin-1 to investigate the expression of DCC receptor and ERK1/2 in patients with ischemic stroke.

In summary, the regulation mechanism of Netrin-1 on the DCC receptor and ERK signaling pathway is not yet known. Based on this, 20 male rats were selected to construct a rat model of MCAO and 10 normal rats were selected as healthy controls (NS). Then, they were divided into the MCAO+Netrin-1 group, MCAO group, and NS group according to the different treatment schemes. The positive expression of Netrin-1 was detected by immunostaining. By comparing the positive expression of Netrin-1, cerebral infarction volume, mNSS, sticker removal test time, cell apoptosis rate, positive expression of DCC, and positive expression of ERK in three kinds of rats, the regulation of Netrin-1 in ischemic stroke and its influence on the DCC/ERK signaling pathway were comprehensively evaluated.

The article "Analysis of Antiapoptosis Effect of Netrin-1 on Ischemic Stroke and Its Molecular Mechanism under Deleted in Colon Cancer/Extracellular Signal-Regulated Kinase Signaling Pathway" was retracted in 2024. Reasons: signs of a paper mill; compromised peer review; unreliable results or conclusions.

## 2. Materials and Methods

### 2.1. Experimental Animals

In this study, 30 clean Sprague-Dawley (SD) rats, aged 10-12 weeks purchased from the xxx University Animal Experiment Center, were selected as the research objects, and 20 of them were selected to construct a rat model of MCAO, and another 10 were selected as healthy controls (NS). Their body weight was between 280 and 300 g, they were raised in a sterile environment at room temperature, the humidity was maintained at about 45%, and food and water were freely available. According to the different treatment regimes, they were divided into the MCAO+Netrin-1 group, MCAO group, and NS group. The experiments were carried out in accordance with the experimental protocol, and the operating procedures were strictly regulated and did not violate ethical requirements.

### 2.2. Construction of a Rat Model of MACO

In this study, a modified Zea-Longa suture method was adopted to prepare a rat model of MCAO. The rats were fasted for 12 hours and then were anesthetized with 20 mg/kg 2% sodium pentobarbital, and their rectal temperature was kept at 37°C. Then, the hair on the rat's neck was shaved, and an approximately 2 cm wound was cut along the midline of the neck. After that, the anterior neck muscle was cut to separate the blistering glands, and the blistering glands were opened and protected with sterile gauze. After the right sternocleidomastoid muscle of the rat was opened, the carotid sheath was found, and the right common carotid artery, external carotid artery, and internal carotid artery were separated in turn. A V-shaped port about 10 mm was cut from the proximal bifurcation of the right common carotid artery, and the prepared thread plug was inserted into the V-shaped port and pushed about 20 mm in the internal carotid artery to the starting position of the anterior cerebral artery. Finally, the thread plug was fixed, the blistering gland was reset, and the skin was sutured.

### 2.3. Virus Striatum Injection of Netrin-1 Overexpression

In this study, all rats were injected with Netrin-1 overexpressing adeno-associated virus vector three weeks before treatment. First, the rats were anesthetized with 20 mg/kg 2% sodium pentobarbital and placed on the brain stereotaxic device in a supine position, and the tip of the steel needle was inserted into the cochlea. Based on the connection between the left and right cochlea in the middle of the head, a 1 cm wound was cut and a small amount of hydrogen peroxide was dripped on the surface of the skull. Then, coordinates of the syringe were adjusted, a hole was drilled vertically from the scalp, and 10 *μ*L of the Netrin-1 overexpression adeno-associated virus vector was slowly injected after the drilling reached a certain depth. After the injection was completed, the brain was sterilized and sutured, and the rats returned to the cage for breeding.

The article "Analysis of Antiapoptosis Effect of Netrin-1 on Ischemic Stroke and Its Molecular Mechanism under Deleted in Colon Cancer/Extracellular Signal-Regulated Kinase Signaling Pathway" was retracted in 2024. Reasons: signs of a paper mill; compromised peer review; unreliable results or conclusions.

### 2.4. Immunohistochemical Staining

The immunohistochemical staining was adopted to detect the positive expression of Netrin-1. After rat brain tissue sections were hydrated and dewaxed, they were soaked in 3% hydrogen peroxide for 20 minutes and washed with PBS (phosphate buffer solution) three times. Then, 10% bovine serum albumin was introduced and the sample was incubated for 30 minutes at 37°C. Then, mouse antiworking solution was included, and the sample was put overnight at 4°C and washed with PBS three times. After that, a biotin-labeled goat anti-mouse secondary antibody working solution was added, the sample was incubated for 20 minutes, and diaminobenzidine (DAB) was used to develop color for 10 minutes. After the color development stopped, the sample was counterstained with hematoxylin for 30 seconds, and the slides were sealed with neutral gum. For the positive evaluation method, 10 field of view areas were selected under a high-definition microscope, the HPIAS-1000 color pathology graphic analysis system produced by Chengdu Powers Technology Co., Ltd. was adopted to automatically count, and the average was taken. For dyeing intensity, 0 points are for no coloring, 1 point for yellow, 2 points for brown, and 3 points for tan. For the proportion of positive cells, 0 points are for less than 10%, 1 point for 10-40%, 2 points for 40-70%, and 3 points for more than 70%. The two were added together for interpretation: 0-1 was negative, 2 was weak positive, 3-4 was positive, and 5-6 was strong positive.

### 2.5. Rat MRI Detection

In this study, MRI was adopted to detect the percentage of rat cerebral infarction volume in the cerebral hemispheres. Before scanning, the rats were subjected to gas anesthesia, and they were fixed on the magnetic resonance head frame. Then, the anesthetic gas was continuously input through the nasal cannula to keep the rat's body temperature at 37°C. T2-weighted turbo positive pressure scan was performed with small animal MRI. After that, images were collected, and ImageJ image processing software was used to calculate the volume of cerebral infarction and the percentage of cerebral hemispheres.

The article "Analysis of Antiapoptosis Effect of Netrin-1 on Ischemic Stroke and Its Molecular Mechanism under Deleted in Colon Cancer/Extracellular Signal-Regulated Kinase Signaling Pathway" was retracted in 2024. Reasons: signs of a paper mill; compromised peer review; unreliable results or conclusions.

### 2.6. Rat Behavior Evaluation

Neurological function evaluation: Modified Neurological Severity Score (mNSS) was adopted to evaluate the neurological function of rats at 0, 1, 3, 5, and 7 days after surgery. The total score was 18 points, and the score was positively correlated with the degree of neurological deficit.

Sensory function evaluation: the sticker removal test was applied to evaluate the sensory function of rats at 0, 1, 3, 5, and 7 days after surgery, the rats were put in a cardboard box, and the wrist of the forelimb was wrapped with a strip of paper. Then, the time the rat used to remove the sticker was recorded, and the average was taken three times. If a rat had not eaten the paper strip for 130 s, the time was recorded as 130 s.

### 2.7. Tunnel Staining Experiment of Rat Brain Tissue

After the paraffin sections of the rat were hydrated and dewaxed, a circle was drawn on the tissue with a histochemical pen, proteinase K solution was added, and the sample was incubated at 37°C for 20 minutes. After the sample was dried, a rupture working solution was added, and the sample was incubated at 25°C for 20 minutes and washed with PBS 3 times. Then, the reagents in the tunnel kit were added to the tissue, and the sample was incubated for 2 hours at 37°C. After that, 3% hydrogen peroxide solution was added to block endogenous peroxidase, and the sample was incubated in the dark for 15 minutes. Then, the reagent converter-POD was introduced after the sample was dried; then, the sample was incubated at 37°C for 30 minutes. Subsequently, DAB color developing solution was added to develop for 15 minutes, and the sample was rinsed with tap water to stop the reaction. Then, the sample was counterstained with hematoxylin for 3 minutes and dehydrated after it returned to blue. Finally, the slides were sealed with neutral gum.

### 2.8. Fluorescence Staining of Rat Brain Tissue Sections

In this study, fluorescent staining was used to detect the expression of DCC and ERK in rats. The cultured cell slides were washed with PBS 3 times, 3 minutes each time. Then, they were fixed with 4% paraformaldehyde for 15 minutes and washed 3 times with PBS. After that, 0.4% Triton X-100 active agent was added, and the sample was incubated at 25°C for 20 minutes and washed 3 times with PBS, 3 minutes each time. Subsequently, goat serum was added, and the sample was incubated for 30 minutes. Then, the corresponding primary antibody working solution was added, and the sample was put at 4°C overnight. Then, a fluorescently labeled secondary antibody working solution was added and the sample was incubated at 25°C for 1 hour. After that, the sample was counterstained with 4′,6-diamidino-2-phenylindole, and finally, the slides were sealed. Finally, the fluorescence intensity of DCC and ERK was observed and calculated under a microscope.

The article "Analysis of Antiapoptosis Effect of Netrin-1 on Ischemic Stroke and Its Molecular Mechanism under Deleted in Colon Cancer/Extracellular Signal-Regulated Kinase Signaling Pathway" was retracted in 2024. Reasons: signs of a paper mill; compromised peer review; unreliable results or conclusions.

### 2.9. Statistical Methods

The data were processed by SPSS19.0, the measurement data were expressed by the mean ± standarddeviation (−*x* ± *s*), and the counting data were expressed by the percentage (%). Pairwise comparison of Netrin-1-positive expression, cerebral infarction volume, mNSS, sticker removal test time, cell apoptosis rate, DCC-positive expression, and ERK-positive expression in the MCAO+Netrin-1 group, MCAO group, and NS group rats was realized by analysis of variance. *P* < 0.05 meant the difference was statistically significant.

## 3. Results

### 3.1. Positive Expression of Netrin-1 in Three Kinds of Rat Brain Tissues

Figure 1 is the comparison of the positive expression rate of Netrin-1 in the brain tissues of three types of rats. It was evident that the positive expression rate of Netrin-1 in the MCAO+Netrin-1 group was 72.46%, that in the MCAO group was 22.04%, and that in the NS group was 19.75%. Among them, the positive expression rate of Netrin-1 in the MCAO+Netrin-1 group was significantly higher than that in the MCAO and NS groups, and the difference was statistically significant (*P* < 0.05).

Figure 2 shows the immunostaining images of Netrin-1 in three rat brain tissues. In Figure 2(a), there were more blue particles and fewer yellow or brown particles, which can be judged as a negative expression of Netrin-1 protein.  Figure 2(b) has a darker degree of staining, with a large number of brown-yellow particles and very few blue particles, which can be judged as a positive expression of Netrin-1 protein.  Figure 2(c) shows a large number of blue particles, almost no yellow or brownish yellow ones, which can be judged as a negative expression of Netrin-1 protein.

### 3.2. The Percentage of Cerebral Infarct Volume in the Cerebral Hemispheres in the Three Groups of Rats

As shown in Figure 3, the percentage of cerebral infarction volume of rats in the cerebral hemisphere in the MCAO+Netrin-1 group was 28.76 ± 2.15%; in the MCAO group, the percentage of rat cerebral infarction volume in the cerebral hemisphere was 45.11 ± 5.85%, and the percentage of cerebral infarction volume in the NS group was 0. Among them, the percentage of cerebral infarction volume of rats in the cerebral hemisphere in the MCAO+Netrin-1 group was significantly higher than that in the MCAO and NS groups, and the difference was statistically significant (*P* < 0.05).  Figure 4 shows MRI images of three types of rat cerebral infarction. It was evident that the cerebral infarction volume of the MCAO group was too large, the cerebral infarction volume of the MCAO group was smaller than that of the MCAO group, and the brain CT image of rats in the NS group was normal.

The article "Analysis of Antiapoptosis Effect of Netrin-1 on Ischemic Stroke and Its Molecular Mechanism under Deleted in Colon Cancer/Extracellular Signal-Regulated Kinase Signaling Pathway" was retracted in 2024. Reasons: signs of a paper mill; compromised peer review; unreliable results or conclusions.

### 3.3. Comparison of Behavioral Performance of the Three Groups of Rats

As shown in Figure 5, the MCAO mNSS and the time spent in the sticker removal test of the rats in the MCAO+Netrin-1 group decreased over time. The MCAO mNSS and the time spent in the sticker removal test of the MCAO+Netrin-1 group were significantly less than those of the MCAO group, and the difference was statistically significant (*P* < 0.05); the MCAO mNSS and the time spent in the sticker removal test of the NS group were always lower than those of the MCAO+Netrin-1 and MCAO groups, and the difference was statistically significant (*P* < 0.05).

### 3.4. Comparison of Cell Apoptosis in Brain Tissue of Three Groups of Rats

As shown in Figure 6, the apoptosis rate of rats in the MCAO+Netrin-1 group was 31.65 ± 1.55%, the percentage of cerebral infarction volume to the cerebral hemisphere in the MCAO group was 48.73 ± 3.74%, and the percentage of cerebral infarction volume to the cerebral hemisphere in the NS group was 7.82 ± 0.97%. The apoptosis rate of rats in the MCAO+Netrin-1 group was significantly lower than that of the MCAO group, and the difference was statistically significant (*P* < 0.05); the apoptosis rate of rats in the NS group was significantly lower than that of the MCAO+Netrin-1 group and the MCAO group, and the difference was statistically significant (*P* < 0.05).  Figure 7 shows the results of apoptosis staining in the brain tissues of the three groups of rats. It was evident that Figure 7(b) has a darker degree of staining with a large number of brown-yellow particles, while in Figures 7(a) and 7(c), there were many blue particles with a lighter degree of coloration.

Note: ^∗^indicated that the difference was statistically significant compared with the NS group (*P* < 0.05); ^#^indicated that the difference was statistically significant compared with the MCAO group (*P* < 0.05).

### 3.5. Comparison of the Positive Expression of DCC in the Brain Tissue of the Three Groups of Rats

As shown in Figure 8, the average fluorescence intensity of DCC of rats in the MCAO+Netrin-1 group was 0.826 ± 0.069, the average fluorescence intensity of DCC of rats in the MCAO group was 0.407 ± 0.038, and the average fluorescence intensity of DCC in the NS group rats was 0.511 ± 0.097. The average fluorescence intensity of DCC in the MCAO+Netrin-1 group was higher than that in the MCAO group, and the difference was statistically significant (*P* < 0.05); the average fluorescence intensity of DCC in the NS group was significantly higher than that of the MCAO+Netrin-1 group and the MCAO group, and the difference was statistically significant (*P* < 0.05).  Figure 9 shows the DCC fluorescence staining results of the three groups of rat brain tissues. It was evident that the fluorescence brightness of Figure 9(a) was significantly better than that of Figures 9(b) and 9(c), and the brightness of Figure 9(b) was the lowest.

The article "Analysis of Antiapoptosis Effect of Netrin-1 on Ischemic Stroke and Its Molecular Mechanism under Deleted in Colon Cancer/Extracellular Signal-Regulated Kinase Signaling Pathway" was retracted in 2024. Reasons: signs of a paper mill; compromised peer review; unreliable results or conclusions.

### 3.6. Comparison of ERK Phosphorylation Levels in Brain Tissue of Three Groups of Rats

As shown in Figure 10, the average fluorescence intensity of DCC of rats in the MCAO+Netrin-1 group was 0.702 ± 0.107, the average fluorescence intensity of DCC of rats in the MCAO group was 0.413 ± 0.082, and the average fluorescence intensity of DCC in the NS group was 0.537 ± 0.059. The p-ERK level in the MCAO+Netrin-1 group was higher than that in the MCAO group, and the difference was statistically significant (*P* < 0.05); the p-ERK level in the NS group was significantly higher than that in the MCAO+Netrin-1 group and the MCAO group, and the difference was statistically significant (*P* < 0.05).  Figure 11 shows the results of p-ERK fluorescence staining in the brain tissues of three groups of rats. It was evident that the fluorescence brightness of p-ERK in Figure 11(a) was significantly better than that in Figures 9(b) and 9(c).

## 4. Discussion

Excitatory toxicity, oxidative stress, and inflammation caused by ischemic stroke onset can cause brain tissue damage and nerve cell apoptosis. Therefore, clinical treatment based on brain tissue and neurons is extremely necessary [13]. In this study, 20 SD rats were selected to construct the MCAO rat model, the other 10 normal rats were taken as healthy controls, and they were divided into the MCAO+Netrin-1 group, MCAO group, and NS group. The results showed that the percentage of cerebral infarction volume in the cerebral hemispheres of the MCAO+Netrin-1 group was significantly higher than that of the MCAO group and the NS group, and the difference was statistically significant (*P* < 0.05), which was similar to the results of Huang et al. [14], indicating that Netrin-1 can effectively reduce the area of cerebral infarction in rats and improve brain tissue damage. The MCAO mNSS and time spent in the sticker removal test in the MCAO+Netrin-1 group were significantly less than those in the MCAO group, and the difference was statistically significant (*P* < 0.05), which was different from the research of Squara et al. [15]. They used mNSS to evaluate the neurological damage of rats, while the sticker removal test was applied to reflect the sensory function of rats, and the results showed that Netrin-1 increasingly improved the behavior of ischemic stroke with time.

The article "Analysis of Antiapoptosis Effect of Netrin-1 on Ischemic Stroke and Its Molecular Mechanism under Deleted in Colon Cancer/Extracellular Signal-Regulated Kinase Signaling Pathway" was retracted in 2024. Reasons: signs of a paper mill; compromised peer review; unreliable results or conclusions.

The rate of apoptosis in rats in the MCAO+Netrin-1 group was significantly lower than that in the MCAO group, and the difference was statistically significant (*P* < 0.05). Studies have shown that Netrin-1 can inhibit tumor diseases. As a result, Netrin-1 can effectively inhibit the apoptosis of rat neuronal cells in ischemic stroke, and its function as a growth factor is also applicable to ischemic stroke disease [16]. The average fluorescence intensity of DCC in the MCAO+Netrin-1 group was higher than that in the MCAO group, and the average fluorescence intensity of the DCC in the NS group was significantly higher than that in the MCAO+Netrin-1 and MCAO groups (*P* < 0.05), which was similar to the results of Rago et al. [17], indicating that the overexpression of Netrin-1 can promote the upregulation of the receptor DCC at the protein level. Therefore, it is speculated that DCC may be involved in the development of ischemia stroke. The p-ERK level of rats in the same MCAO+Netrin-1 group was higher than that in the MCAO group, and the p-ERK level of rats in the NS group was significantly higher than that in the MCAO+Netrin-1 group and the MCAO group (*P* < 0.05), which indicated that the overexpression of Netrin-1 can increase the phosphorylation level of ERK, and it is speculated that the EPK signaling pathway may be involved in the antiapoptotic effect of Netrin-1.

## 5. Conclusion

In this study, 20 SD rats were selected to construct a MCAO rat model, another 10 normal rats were taken as healthy controls, and they were divided into the MCAO+Netrin-1 group, MCAO group, and NS group according to the different treatment schemes. It was found that Netrin-1 can effectively reduce brain tissue damage in rats with ischemic stroke, improve the neurological and sensory functions of rats, and also effectively inhibit neuronal cell apoptosis, and Netrin-1 can promote DCC expression and ERK phosphorylation, and EPK signaling pathway may be involved in the antiapoptotic effect of Netrin-1. However, the sample size of rats selected in this study is small, and the DNA repair protein and mitochondrial damage are not discussed. The subsequent research will increase the number of animal samples for further analysis. In conclusion, the results of this study provide a theoretical basis for the application of Netrin-1 in ischemic stroke disease.

## Figures and Tables

**Figure 1:** Comparison of the positive expression rate of Netrin-1 protein in the brain tissues of three types of rats. Note: ^∗^meant that the difference was statistically significant compared to the MCAO+Netrin-1 group of rats (*P* < 0.05).

The article "Analysis of Antiapoptosis Effect of Netrin-1 on Ischemic Stroke and Its Molecular Mechanism under Deleted in Colon Cancer/Extracellular Signal-Regulated Kinase Signaling Pathway" was retracted in 2024. Reasons: signs of a paper mill; compromised peer review; unreliable results or conclusions.

**Figure 2:** Immunostaining results of Netrin-1 protein of three kinds of rat brain tissue. Note: (a) the rats in the MCAO+Netrin-1 group; (b) the rats in the MCAO group; (c) the rats in the NS group.

**Figure 3:** The percentage of cerebral infarct volume in the cerebral hemisphere of three kinds of rats. Note: ^∗^meant that the difference was statistically significant compared to the MCAO+Netrin-1 group of rats (*P* < 0.05).

**Figure 4:** MRI images of cerebral infarction of three types of rats. Note: (a) the rats in the MCAO+Netrin-1 group; (b) the rats in the MCAO group; (c) the rats in the NS group.

**Figure 5:** Comparison of the behavioral performance of three groups of rats. Note: (a) the score of neurological function in rats; (b) the time spent in the sticker removal test. ^∗^Indicated that the difference was statistically significant compared to the NS group of rats (*P* < 0.05); ^#^indicated that the difference was statistically significant compared to the MCAO group of rats (*P* < 0.05).

**Figure 6:** Comparison of cell apoptosis in brain tissues of three groups of rats.

**Figure 7:** Apoptosis staining results of brain cells in three groups of rats. Note: (a) the MCAO+Netrin-1 group of rats; (b) the MCAO group of rats; (c) the NS group of rats.

**Figure 8:** Comparison of brain DCC-positive expression of three groups of rats. Note: ^∗^indicated that the difference was statistically significant compared with the NS group (*P* < 0.05); ^#^indicated that the difference was statistically significant compared with the MCAO group (*P* < 0.05).

**Figure 9:** Fluorescence staining results of DCC in the brain tissue of three groups of rats. Note: (a) the rats in the MCAO+Netrin-1 group; (b) the rats in the MCAO group; (c) the rats in the NS group.

**Figure 10:** Comparison of brain p-ERK of three groups of rats. Note: ^∗^indicated that the difference was statistically significant compared with the NS group (*P* < 0.05); ^#^indicated that the difference was statistically significant compared with the MCAO group (*P* < 0.05).

**Figure 11:** Results of p-ERK fluorescence staining of brain tissue sections in three groups of rats. Note: (a) the rats in the MCAO+Netrin-1 group; (b) the rats in the MCAO group; (c) the rats in the NS group.

## Data Availability

All data, models, and code generated or used during the study appear in the submitted article.
